RETRACTED

# Deep Fractional Max Pooling Neural Network for COVID-19 Recognition

**DOI:** 10.3389/fpubh.2021.726144

**Published:** 2021-08-10

**Authors:** Shui-Hua Wang, Suresh Chandra Satapathy, Donovan Anderson, Shi-Xin Chen, Yu-Dong Zhang

**Affiliations:** ^1^School of Mathematics and Actuarial Science, University of Leicester, Leicester, United Kingdom; ^2^School of Computer Engineering, KIIT Deemed to University, Bhubaneswar, India; ^3^Nursing Department, The Fourth People's Hospital of Huai'an, Huai'an, China; ^4^School of Informatics, University of Leicester, Leicester, United Kingdom

**Keywords:** convolutional neural network, fractional max pooling, data augmentation, COVID-19, average pooling, model averaging

## Abstract

**Aim:** Coronavirus disease 2019 (COVID-19) is a form of disease triggered by a new strain of coronavirus. This paper proposes a novel model termed “deep fractional max pooling neural network (DFMPNN)” to diagnose COVID-19 more efficiently.

**Methods:** This 12-layer DFMPNN replaces max pooling (MP) and average pooling (AP) in ordinary neural networks with the help of a novel pooling method called “fractional max-pooling” (FMP). In addition, multiple-way data augmentation (DA) is employed to reduce overfitting. Model averaging (MA) is used to reduce randomness.

**Results:** We ran our algorithm on a four-category dataset that contained COVID-19, community-acquired pneumonia, secondary pulmonary tuberculosis (SPT), and healthy control (HC). The 10 runs on the test set show that the micro-averaged F1 (MAF) score of our DFMPNN is 95.88%.

**Discussions:** This proposed DFMPNN is superior to 10 state-of-the-art models. Besides, FMP outperforms traditional MP, AP, and L2-norm pooling (L2P).

## Introduction

Coronavirus disease 2019 (COVID-19) is a form of disease triggered by a new strain of coronavirus. “CO” stands for corona; “VI” virus; and “D,” disease. Until 28 June 2021, COVID-19 caused more than 181.437 million confirmed cases and over 3.929 million deaths. The pie chart of the top 10 countries with new cases, new death tolls, cumulated cases, and cumulated death tolls is displayed in Figure 1.

**Figure 1:** Pie charts of the top 10 countries. **(A)** New cases, **(B)** new death tolls, **(C)** cumulated cases, and **(D)** cumulated death tolls.

To effectively diagnose COVID-19, there exist two types of methods: (i) polymerase chain reaction (PCR), particularly real-time reverse-transcriptase PCR (rRT-PCR) with nasopharyngeal swab samples to test the existence of RNA fragments (1); and (ii) chest imaging (CI) examines the evidence of COVID-19 in the lung.

The rRT-PCR is commonly used nowadays, but it has three shortcomings: (i) It has to wait for a few days to get the results; (ii) The samples are easily contaminated by the environment; (iii) Its performances on COVID-19 variants (2) are still under investigation.

RETRACTED

On the contrary, CI diagnosis has quite a few advantages compared to rRT-PCR (3). (i) Chest imaging is able to detect conclusive evidence—lesions of lungs where “ground-glass opacity (GGO)” patches are observed to distinguish COVID-19 from healthy people. (ii) Chest imaging provides an instant result as soon as imaging is complete. (iii) The previous study shows that chest computed tomography (CCT), one CI approach, can detect 97% of COVID-19 infections (4).

At present, there exist three styles of CI approaches: (i) chest X-ray, (ii) chest CT, and (iii) chest ultrasound. Among all three styles of CI approaches, CCT is capable of providing finer resolution than the other two styles (chest X-ray and chest ultrasound), granting visualization of exceptionally small nodules in the lung, and displaying the realistic three-dimensional imaging of the chest (5). Some COVID-19 lesions are clearly observed in CCT, while they appear opaque in the other two CI approaches (chest X-ray and chest ultrasound) (6).

However, manual labeling on CCT images by human experts is tedious, onerous, labor-intensive, and time-consuming. In addition, the labeling performances are easily affected by inter-expert and intra-expert factors (e.g., emotion, lethargy, tiredness, etc.). Furthermore, early-stage lesions are small and look similar to nearby healthy tissues (7), making them more difficult to measure. Thus, those lesions are potentially ignored by human experts.

Therefore, scholars nowadays favor using artificial intelligence (AI) and modern deep learning (DL) to assist radiologists in recognizing COVID-19. Yao (8) proposed a wavelet entropy biogeography-based optimization (WEBBO) method for COVID-19 diagnosis. Wu (9) presented three-segment biogeography-based optimization (3SBBO) for recognizing COVID-19 patients. Wang et al. (10) presented a DeCovNet. Their accuracy achieved 90.1%. El-kenawy et al. (11) presented a novel feature selection voting classifier (FSVC) method for COVID-19 classification. Yu et al. (12) presented a light-weight GoogleNet-COD method (abbreviated as GN-COD in this paper) to detect COVID-19. Chen (13) designed a gray-level co-occurrence matrix and support vector machine (GLCMSVM) method to classify COVID-19 images. Satapathy (14) presented a five-layer deep convolutional neural network (DCNN). In their paper, the authors presented stochastic pooling to replace traditional pooling methods. Cohen et al. (15) proposed a COVID severity score network (CSSN). FCONet Ko et al. (16) proposed a fast-track COVID-19 network (FCONet). Li et al. (17) presented a COVID-19 detection neural network (COVNet). Cheng (18) proposed a PatchShuffle stochastic pooling neural network (PSSPNN). Ten runs based on training-set split validation showed their method arrived at a micro-averaged F1 (MAF) score of 95.79%. Hammoudi et al. (19) investigated DL methods for analyzing query chest X-ray images automatically. Nigam et al. (20) tested five pretrained models: VGG16, DenseNet121, Xception, NASNet, and EfficientNet.

RETRACTED

From the above recent COVID-19 literature, we can observe DL, generally, can obtain better performances than traditional AI methods. To further improve the COVID-19 recognition performance, this study suggests harnessing fractional max-pooling (FMP) to replace traditional max pooling (MP)/average pooling (AP). Thus, we propose a novel deep fractional max pooling neural network (DFMPNN) to help automatic COVID-19 recognition. Our contributions entail the following four aspects:

(i) The FMP is introduced to replace traditional MP and AP.
(ii) A new “DFMPNN” model is proposed.
(iii) Multiple-way data augmentation (DA) is harnessed to aid the network in avoiding overfitting.
(iv) DFMPNN is proven to yield better results than 10 state-of-the-art COVID-19 recognition methods.

## Dataset

Four types (*k* = 1, 2, 3, *and* 4) of CCT are obtained and used from (18): (i) COVID-19 positive patients; (ii) community-acquired pneumonia (shortened as CAP); (iii) secondary pulmonary tuberculosis (SPT); (iv) healthy control (HC).


(1) $$Class=\{\begin{array}{c} Covid-19\\ CAP\\ SPT\\ HC \end{array}\;,if\;k=\{\begin{array}{c} 1\\ 2\\ 3\\ 4 \end{array}$$

For *o*-th subject, *m*(*o*) slices of CCT are chosen *via* slice level selection (SLS). For HC subjects, any slices within the 3D image are randomly chosen. For the three diseased groups (COVID-19, CAP, and SPT), the slices displaying the largest number of lesions and size are chosen.

The slice-to-subject ratio (STSR) per class $\bar{m}\;\left(k\right)$is defined as


(2) $$\begin{array}{l} \bar{m}\;\left(k\right)=\frac{m_{S}\;\left(k\right)}{m_{P}\left(k\right)},k=1,\;2,\;3,\;and\;4 \end{array}$$

where *m*_*S*_(*k*) means the number of slices per class *via* the SLS, and, *m*_*P*_(*k*), the number of patients per class. The overall STSR is defined as


(3) $$\begin{array}{l} \bar{m}=\frac{\sum_{k=1}^{4}m_{S}\left(k\right)}{\sum_{k=1}^{4}m_{P}\left(k\right)} \end{array}$$

Five hundred and twenty-one subjects and 1,164 slice images were enrolled and extracted in (18). Table 1 lists the demographics of the four-class cohort. Meanwhile, the values of triplets $\left[\bar{m}\left(k\right),m_{P}\left(k\right),{and\;m}_{S}\left(k\right)\right]$of each class are displayed. From Table 1, we can observe the overall STSR $\bar{m}=\;2.23$.

RETRACTED

**Table 1:** Subjects and images of four categories.

*k*	$\bar{m}\left(k\right)$	*m_P_*(*k*)	*m_S_*(*k*)
1	2.27	125	284
2	2.28	123	281
3	2.18	134	293
4	2.20	139	306
Overall	2.23	521	1164

Three experienced radiologists—one senior: $M_{3\;}$and two juniors: $M_{1}$ and $M_{2}$–were convened to curate all the images. Let *b*_*C*_ mean one CCT scan and *l*_*A*_ the labeling of each individual radiologist. The concluding labeling $l_{A}^{F}$ of the CCT scan *b*_*C*_ is written as:


(4) $$l_{A}^{F}\left[b_{C}\right]=\{\begin{array}{c} l_{A}\left[{ℳ}_{1},b_{C}\right]\;l_{A}\left[{ℳ}_{1},b_{C}\right]==l_{A}\left[{ℳ}_{2},b_{C}\right]\\ h_{MAV}\left[l_{A}^{All}\left(b_{C}\right)\right]\;otherwise \end{array}$$

where *h*_*MAV*_ denotes majority voting (MAV) function; $l_{A}^{All}$, the labeling of all three radiologists, *viz*.,


(5) $$\begin{array}{l} l_{A}^{All}\left(b_{C}\right)=\left[l_{A}\left(M_{1},b_{C}\right),l_{A}\left(M_{2},b_{C}\right),l_{A}\left(M_{3},b_{C}\right)\right] \end{array}$$

The above two formulas indicate that in cases of disagreement between the analyses of two junior radiologists $\left(M_{1},M_{2}\right)$, a senior radiologist $\left(M_{3}\right)\;$is consulted to reach a MAV-type consensus.

## Methodology

### Preprocessing

Table 2 presents the abbreviations and corresponding definitions. Let the raw dataset be symbolized as *F*_*A*_, each slice be symbolized as *f*_*a*_, and the number of total slices of all four classes be |*F*|, we have


(6) $$\begin{array}{l} F_{A}=\left\{f_{a}\left(i\right),i=1,2,\cdots \;,|F|\right\} \end{array}$$

**Table 2:** Abbreviation and full name.

**Abbreviation**	**Definition**
PCR	Polymerase chain reaction
CI	Chest imaging
rRT-PCR	Real-time reverse-transcriptase PCR
CCT	Chest computed tomography
AI	Artificial intelligence
DFMPNN	Deep fractional max pooling neural network
DL	Deep learning
FMP	Fractional max pooling
CAP	Community-acquired pneumonia
SPT	Secondary pulmonary tuberculosis
HC	Healthy control
SLS	Slice level selection
STSR	Slice-to-subject ratio
MAV	Majority voting
HS	Histogram stretching
DCR	Data compression ratio
SSR	Space-saving ratio
FM	Feature map
FMP	Fractional max pooling
NWL	Number of weighted layers
HS	Hyperparameer setting
MA	Model averaging
DA	Data augmentation
TCM	Test confusion matrix
L2P	L2-norm pooling
MP	Max pooling
AP	Average pooling
MAF	Micro-averaged F1

The size of each image is


(7) $$\begin{array}{l} h_{size\;}\left[f_{a}\left(i\right)\right]=W_{F_{A}}\times H_{F_{A}}\times 3 \end{array}$$

where (*W*_*F*_*A*__, *H*_*F*_*A*__) means the maximum values of width and height to the image set *F*_*A*_. *h*_*size*_ is the size function. Figure 2 portrays the pipeline for preprocessing. Here, *W*_*F*_*A*__ = *H*_*F*_*A*__ = 1, 014.

RETRACTED

**Figure 2:** A diagram of preprocessing for each slice.

First, the color CCT images are converted into gray scale by retaining the luminance channel and obtaining the gray scale (21). The grayscaled data set is symbolized as *F*_*B*_ = {*f*_*b*_(*i*), *i* = 1, 2, ⋯ , |*F*|}. If (*v*_*r*_, *v*_*g*_, *v*_*b*_) denotes the values of red, green, and blue color channels, the grayscaled image is calculated as


(8) $$\begin{array}{l} f_{b}\left(i\right)=0.2989\times v_{r}\;\left[f_{a}\left(i\right)\right]+0.5870\times v_{g}\left[f_{a}\left(i\right)\right]\\ \;+0.1140\times v_{b}\left[f_{a}\left(i\right)\right] \end{array}$$

Second, the histogram stretching (HS) is harnessed to increase the contrast of all images {*f*_*b*_(*i*)}. Take the *i*-th image *f*_*b*_(*i*) as an instance; its image-wise minimum grayscale value $f_{b}^{l}\left(i\right)\;$is calculated as:


(9) $$\begin{array}{l} f_{b}^{l}\left(i\right)=\overset{W_{F_{B}}}{\underset{w=1}{\min}}\overset{H_{F_{B}}}{\underset{h=1}{\min}}f_{b}\left(i|w,h\right) \end{array}$$

The image-wise maximum grayscale values $f_{b}^{h}\left(i\right)\;$is calculated as:


(10) $$\begin{array}{l} f_{b}^{h}\left(i\right)=\overset{W_{F_{B}}}{\underset{w=1}{\max}}\overset{H_{F_{B}}}{\underset{h=1}{\max}}f_{b}\left(i|w,h\right) \end{array}$$

Here, (*w, h*) means the index of width and height directions along with the image *f*_*b*_(*i*), respectively. (*W*_*F*_*B*__, *H*_*F*_*B*__) means the maximum values of width and height to the image set *F*_*B*_. The histogram stretched image set *F*_*C*_ = {*f*_*c*_(*i*), *i* = 1, 2, ⋯ , |*F*|} is calculated as:


(11) $$\begin{array}{l} f_{c}\left(i\right)=\frac{f_{b}\left(i\right)-f_{b}^{l}\left(i\right)}{f_{b}^{h}\left(i\right)-f_{b}^{l}\left(i\right)} \end{array}$$

Third, cropping is performed to remove (i) the checkup bed at the bottom area, (ii) the texts at the margin regions, and (iii) the ruler along the right-side and bottom areas. Each image in the cropped dataset *F*_*D*_ = {*f*_*d*_(*i*), *i* = 1, 2, ⋯ , |*F*|} is yielded by


(12) $$\begin{array}{l} f_{d}\left(i\right)=f_{c}\left(i;w,h\right),w\in \left[c_{1},W_{F_{C}}-c_{2}\right],h\in \left[c_{3},H_{F_{C}}-c_{4}\right] \end{array}$$

where (*W*_*F*_*C*__, *H*_*F*_*C*__) means the maximum values of width and height to the image set *F*_*C*_. (*c*_1_, *c*_2_, *c*_3_, *c*_4_) means pixels to be cropped from four directions of the left, right, top, and bottom, respectively (unit: pixel).

Fourth, each image in *F*_*D*_ is downsampled to a size of [*W*_*F*_*E*__, *H*_*F*_*E*__], obtaining the resized image set *F*_*E*_ = {*f*_*e*_(*i*), *i* = 1, 2, ⋯ , |*F*|} as


(13) $$\begin{array}{l} f_{e}\left(i\right)=h_{res}\left[f_{d}\left(i\right);\left(W_{F_{E}},H_{F_{E}}\right)\right] \end{array}$$

where *h*_*res*_ stands for the resizing function. In this study, *W*_*F*_*E*__ = *H*_*F*_*E*__ = 256.

RETRACTED

Figure 3 displays exemplar images of the four classes, where three are diseased and one is healthy. The meaning of *k* can be found at Table 1. The original size of each image in *F*_*A*_ is *W*_*F*_*A*__ × *H*_*F*_*A*__ × 3, and the final preprocessed image in *F*_*E*_ is *W*_*F*_*E*__ × *H*_*F*_*E*__. The data compression ratio (DCR) (22) value *v*_*DCR*_ can be calculated as


(14) $$\begin{array}{l} v_{DCR}=\frac{W_{F_{A}}\times H_{F_{A}}\times 3}{W_{F_{E}}\times H_{F_{E}}}=\frac{1024^{2}\times 3}{256^{2}}=48 \end{array}$$

**Figure 3:** Samples of four categories (*k* = 1, 2, 3, and 4). **(A)** *k* = 1, COVID-19, **(B)** *k* = 2, CAP, **(C)** *k* = 3, SPT, and **(D)** *k* = 4, HC.

The space-saving ratio (SSR) value *v*_*SSR*_can be calculated as.


(15) $$\begin{array}{l} v_{SSR}=1-\frac{W_{F_{E}}\times H_{F_{E}}}{W_{F_{A}}\times H_{F_{A}}\times 3}=1-\frac{256^{2}}{1024^{2}\times 3}=97.92\% \end{array}$$

### Traditional Pooling

Pooling is necessary to reduce the size of the feature map (FM) (23), which is generated after the convolution layer. Suppose, the input FM is with the size of *N*_*in*_ × *N*_*in*_, and the output FM is *N*_*out*_ × *N*_*out*_. Usually, *N*_*out*_ < *N*_*in*_. In another sense, the pooling divides the input FM into $N_{out}^{2}\;$pooling regions {*P*_*ij*_}


(16) $$\begin{array}{l} P_{ij}\subset {\left\{1,2,\ldots ,N_{in}\right\}}^{2},i\in \left[1,\ldots ,N_{out}\right],j\in \left[1,\ldots ,N_{out}\right] \end{array}$$

The output is


(17) $$\begin{array}{l} Output_{ij}=\underset{\left(k,l\right)\in P_{ij}}{h_{pool}}Input_{kl} \end{array}$$

where *h*_*pool*_ is different pooling function, such as max function in MP or average function in AP (24). There are also more complicated pooling functions, such as the stochastic function (25) and rank-based functions.

Traditional regular pooling methods with astride (α) of 2 are analyzed. For non-overlapping, we have


(18) $$\{\begin{array}{c} \begin{array}{c} N_{in}=2N_{out}\\ P_{ij}=\left\{2i-1,2i\right\}\times \left\{2j-1,2j\right\} \end{array} \end{array}\;,\;disjoint$$

For overlapping, we have


(19) $$\{\begin{array}{c} \begin{array}{c} N_{in}=2N_{out}+1\\ P_{ij}=\left\{2i-1,2i,2i+1\right\}\times \left\{2j-1,2j,2j+1\right\} \end{array} \end{array},overlapping$$

The pooling regions of both cases are portrayed in Figure 4. The red, green, yellow, and blue rectangles represent the four steps of both pooling procedures. In either non-overlapping or overlapping cases, we can observe


(20) $$\begin{array}{l} \frac{N_{in}}{N_{out}}\approx 2,\;if\;\alpha =2 \end{array}$$

**Figure 4:** Traditional regular pooling with a stride of 2. **(A)** Disjoint. **(B)** Overlapping.

RETRACTED

Thus, the spatial size of FM halves in size with each pooling layer. This halving brings a by-product of discarding 1 − (0.5)^2^ = 75% information of the previous FM. The rapid reduction may worsen the performance.

### Fractional Max Pooling

Therefore, Graham (26) proposed a novel fractional max pooling (FMP), i.e., α × α MP, where α is allowed to take non-integer values. In their paper, they set


(21) $$\begin{array}{l} FMP:\frac{N_{in}}{N_{out}}\approx \sqrt[{n}]{2} \end{array}$$

So this can help make the pooling *n* times slower than the regular 2 × 2 pooling. FMP has been extended to new models, such as bi-linearly weighted FMP (27) and shallow and wide FMP (28).

Assume ${\left(a_{i}\right)}_{i=1}^{N_{out}+1}$ and ${\left(b_{i}\right)}_{i=1}^{N_{out}+1}$ are two increasing sequences of integers with *N*_*out*_ numbers, staring at 1 and ending with 1 + *N*_*in*_. Also, all increments equal to either 1 or 2. That is


(22) $$\{\begin{array}{c} a_{1}=1\\ a_{N_{out}+1}=1+N_{in}\\ a_{i+1}-a_{i}\in \left\{1,2\right\} \end{array}$$

The pooling regions can be formulated as:


(23) $$\begin{array}{l} P_{Ij}=\left[a_{i-1},a_{i}-1\right]\times \left[b_{j-1},b_{j}-1\right],\;disjoint \end{array}$$

(24) $$\begin{array}{l} P_{Ij}=\left[a_{i-1},a_{i}\right]\times \left[b_{j-1},b_{j}\right],\;overlapping \end{array}$$

In this study, we choose disjoint type FMP. We also tested overlapping FMP; the computation burden increases, but the performance does not improve. Figure 5A shows a square grid where *N*_*in*_ = 30. Figures 5B–D shows the FMP results according to α = 1.4, 1.5, and 1.6, respectively. The corresponding *N*_*out*_ = 21, 20, and 19, respectively. Finally, Figure 5E displays the result with α = 2, which corresponds to the regular 2 × 2 pooling where the output *N*_*out*_ = 15.

**Figure 5:** Illustration of FMP (This figure may make you uncomfortable). **(A)** Square Grid (30 × 30), **(B)** α = 1.4, **(C)** α = 1.5, **(D)** α = 1.6, and **(E)** α = 2.

### Deep Fractional Max Pooling Neural Network

We built a 12-layer DFMPNN from scratch. Its structure is itemized in Table 3. Here, NWL represents the number of weighted layers and HS hyperparameter setting. Transfer learning, such as ResNet-50 (29), may help quickly build the network. In our study, we find ResNet-50 and other pretrained models do not provide competitive performances as building networks from scratch, which is coherent with the reports in (20).

RETRACTED

**Table 3:** Structure of proposed 12-layer DFMPNN.

**Index**	**Name**	**NWL**	**HS**	**Size of FM**
1	Input			256 × 256 × 1
2	Conv-1	1	32, 5 × 5 *s* = 2	128 × 128 × 32
3	FMP-1		$\alpha =\sqrt{2}$	91 × 91 × 32
4	Conv-2	1	64, 3 × 3	91 × 91 × 64
5	FMP-2		$\alpha =\sqrt{2}$	64 × 64 × 64
6	Conv-3	1	96, 3 × 3	64 × 64 × 96
7	FMP-3		$\alpha =\sqrt{2}$	45 × 45 × 96
8	Conv-4	1	128, 3 × 3	45 × 45 × 128
9	FMP-4		$\alpha =\sqrt{2}$	32 × 32 × 128
10	Conv-5	1	160, 3 × 3	32 × 32 × 160
11	FMP-5		$\alpha =\sqrt{2}$	23 × 23 × 160
12	Conv-6	1	192, 3 × 3	23 × 23 × 192
13	FMP-6		$\alpha =\sqrt{2}$	16 × 16 × 192
14	Conv-7	1	224, 3 × 3	16 × 16 × 224
15	FMP-7		$\alpha =\sqrt{2}$	11 × 11 × 224
16	Conv-8	1	256, 3 × 3	11 × 11 × 256
17	FMP-8		$\alpha =\sqrt{2}$	8 × 8 × 256
18	Conv-9	1	288, 3 × 3	8 × 8 × 288
19	FMP-9		$\alpha =\sqrt{2}$	6 × 6 × 288
20	Conv-10	1	320, 3 × 3	6 × 6 × 320
21	FMP-10		$\alpha =\sqrt{2}$	4 × 4 × 320
22	Flatten			1 × 1 × 5120
23	FCL-1	1	200 × 5120, 200 × 1	1 × 1 × 200
24	FCL-2	1	4 × 200, 4 × 1	1 × 1 × 4
25	Softmax			1 × 1 × 4

Figure 6 shows the FM of all layers of this DFMPNN. Since our network is deep, we show Layer 1 to Layer 13 at Figure 6A and Layer 13 to Layer 25 at Figure 6B. Note that $\frac{128}{91}=1.4066$, $\frac{91}{64}=1.421$, $\frac{64}{45}=1.422$, $\frac{45}{32}=1.4062$, $\frac{32}{23}=1.391$, $\frac{23}{\;16}=1.4375$, $\;\frac{16}{11}=1.454$ $\frac{11}{8}=1.3750$, $\frac{8}{6}=1.3333$, $\frac{6}{4}=1.5000$. All the values approximate to $\sqrt{2}=1.414$2.

**Figure 6:** FM of proposed DFMPNN. **(A)** From layer 1 to Layer 13. **(B)** From Layer 13 to Layer 25.

Model averaging(MA) (30) is a robust way to handle the randomness and uncertainty in this proposed DFMPNN model, in which the random sequences {*a*_*i*_} and {*b*_*i*_} are generated differently at each run. Therefore, this network can be easily implemented multiple times, and thus making an ensemble of those implementations (31). That is, the different pooling-region setting of each implementation defines a different member of the ensemble. The MA can help DFMPNN get better results. For a given test image, if we implement *T* tests, the MAV of the *T*tests will be used as the final prediction.

### Multiple-Way Data Augmentation

To alleviate the overfitting and coping with the small-size dataset problem, we used the 18-way DA in (32). In their paper, *X*_1_ = 9 different DA methods were used on both the raw image *r*(*i*) and its horizontally mirrored image *r*^*hm*^(*i*). The *X*_1_DAs are rotation, Gaussian noise, Gamma correction, random translation, vertical shear, salt-and-pepper noise, speckle noise, horizontal shear, and scaling, shown in Figure 7.

RETRACTED

**Figure 7:** A diagram of 18-way DA.

Suppose, the raw image is *r*(*i*) and the number of DA methods *X*_1_. Let *x* be the index of DA, and **K**_*x*_, *x* = 1, …, *X*_1_ be each DA operation; we have:

**Step 1**, *X*_1_ geometric/photometric/noise-injection DA transforms are utilized on raw image *r*(*i*). Thus, we have *X*_1_ augmented datasets on raw image *r*(*i*) as


(25) $$\begin{array}{l} {\text{K}}_{x}\left[r\left(i\right)\right],x=1,\ldots ,X_{1} \end{array}$$

Note, each DA operations **K**_*x*_ will yield *X*_2_ new images:


(26) $$\begin{array}{l} |{\text{K}}_{x}\left[r\left(i\right)\right]|=X_{2}. \end{array}$$

**Step 2**, horizontally mirrored image*r*^*hm*^(*i*) is generated *via* the horizontally mirrored function *h*_*m*_,


(27) $$\begin{array}{l} r^{hm}\left(i\right)=h_{m}\left[r\left(i\right)\right] \end{array}$$

**Step 3**, all the *X*_1_ different DA methods are performed on the horizontally mirrored image *r*^*hm*^(*i*), and generate *X*_1_ new datasets as


(28) $$\{\begin{array}{c} K_{x}\left[r^{hm}\left(i\right)\right],x=1,\cdots ,X_{1}\\ \left|K_{x}\left[r^{hm}\left(i\right)\right]\right|=X_{2},x=1,\ldots ,X_{1} \end{array}$$

**Step 4**, the *r*(*i*), *r*^*hm*^(*i*), **K**_*x*_[*r*(*i*)], *x* = 1, …, *X*_1_, and ${\text{K}}_{x}\left[r^{hm}\left(i\right)\right],x=1,\cdots \;,X_{1}$ are combined *via* the concatenation function *h*_*co*_. That is, one raw training image *r*(*i*) will generate to an enhanced dataset 𝔻(*i*):


(29) $$r\left(i\right)\mapsto 𝔻\left(i\right)=h_{co}\left\{\begin{array}{cc} r\left(i\right) & r^{hm}\left(i\right)\\ \underset{\cdots }{\underset{\underset{X_{2}}{\underset{︸}{10mm}}}{K_{1}\left[r\left(i\right)\right]}} & \underset{\cdots }{\underset{\underset{X_{2}}{\underset{︸}{10mm}}}{K_{1}[r^{hm}\left(i\right)]}}\\ \underset{\underset{X_{2}}{\underset{︸}{10mm}}}{K_{X1}\left[r\left(i\right)\right]} & \underset{\underset{X_{2}}{\underset{︸}{10mm}}}{K_{1}[r^{hm}\left(i\right)]} \end{array}\right\}$$

Let *X*_3_ represent the augmentation factor, i.e., the number of elements in the enhanced dataset 𝔻(*i*),; we have


(30) $$\begin{array}{l} X_{3}=\frac{\left|𝔻\left(i\right)\right|}{\left|r\left(i\right)\right|}=\frac{\left(1+X_{1}\times X_{2}\right)\times 2}{1}=2\times X_{1}\times X_{2}+2 \end{array}$$

Finally, Table 4 shows the pseudocode of 18-way DA.

**Table 4:** Pseudocode of 18-way DA.

**Import**	**Raw image *r*(*i*)**.
Step 1.1	*X*_1_ geometric/photometric/noise-injection DA transforms are utilized on raw image *r*(*i*).
Step 1.2	We obtain *K*_*x*_[*r*(*i*)], *x* = 1, …, *X*_1_ datasets. See Equation (25).
Step 1.3	Each dataset contains *X*_2_ images. See Equation (26).
Step 2	A horizontal mirror image is generated as $r^{hm}\left(i\right)=h_{m}\left[r\left(i\right)\right]$. See Equation (27).
Step 3.1	*X*_1_ DA transforms are utilized on thehorizontally mirrored image *r*^*hm*^(*i*).
Step 3.2	We obtain $K_{x}\left[r^{hm}\left(i\right)\right],x=1,\cdots \;,X_{1}$ datasets. Each dataset contains *X*_2_ images. See. Equation (28).
Step 4	The *r*(*i*), *r*^*hm*^(*i*), *K*_*x*_[*r*(*i*)], *x* = 1, …, *X*_1_, and $K_{x}\left[r^{hm}\left(i\right)\right],x=1,\cdots \;,X_{1}$are combined to form a new enhanced dataset *D*(*i*). See Equation (29).
Output	Enhanced dataset *D*(*i*). Its number of images is *X*_3_ = 2 × *X*_1_ × *X*_2_ + 2. See Equation (30).

RETRACTED

### Implementation and Measures

Table 5 lists the non-test and test sets of each category. The whole dataset is symbolized as *U*contains four non-overlapping categories *U* = {*U*_*k*_} = {*U*_1_, *U*_2_, *U*_3_, *U*_4_}. See Table 1 to check the meanings of each class {*k*}. For each category, the set *U* will be split into the non-test set and test set $U_{k}\to \left\{U_{k}^{ntest},U_{k}^{test}\right\},k=1,\ldots ,4$. The non-test set will cover 80% of the total set, and the test set will cover 20% of the total set.


(31) $$\begin{array}{l} U=\left[\begin{array}{c} U_{1}\\ U_{2}\\ U_{3}\\ U_{4} \end{array}\right]=\left[\begin{array}{cc} U^{ntest} & U^{test} \end{array}\right]=\left[\begin{array}{cc} U_{1}^{ntest} & U_{1}^{test}\\ U_{2}^{ntest} & U_{2}^{test}\\ U_{3}^{ntest} & U_{3}^{test}\\ U_{4}^{ntest} & U_{4}^{test} \end{array}\right] \end{array}$$

**Table 5:** Splitting setting of our dataset.

**Category (*k)***	**Non-test (80%)**	**Test (20%)**	**Total (100%)**
*k* = 1	$|U_{1}^{ntest}|=227$	$|U_{1}^{test}|=57$	|*U*_1_| = 284
*k* = 2	$|U_{2}^{ntest}|=225$	$|U_{2}^{test}|=56$	|*U*_2_| = 281
*k* = 3	$|U_{3}^{ntest}|=234$	$|U_{3}^{test}|=59$	|*U*_3_| = 293
*k* = 4	$|U_{4}^{ntest}|=245$	$|U_{4}^{test}|=61$	|*U*_4_| = 306

The experiment consists of two phases. At Phase I “Validation,” 10-fold cross-validation is harnessed for validation on the non-test set, for the aim of selecting the best hyperparameters and best network structure. The 18-way DA is utilized on the training set.

At Phase II “Test,” our model is trained, using the non-test set *U*^*ntest*^*Q*^*t*^ times with (i) different initial seeds and (ii) the best hyperparameters/network structure obtained at Phase I. We attained the test results over the test set *U*^*test*^. Once combining the *Q*^*t*^ runs, a summation of the test confusion matrix (TCM) *E*^*t*^ is obtained.

The ideal TCM is a diagonal matrix with the form of


(32) $$\begin{array}{l} E_{ideal}^{t}=Q^{t}\times \left[\begin{array}{cccc} \left|U_{1}^{test}\right| & 0 & 0 & 0\\ 0 & \left|U_{2}^{test}\right| & 0 & 0\\ 0 & 0 & \left|U_{3}^{test}\right| & 0\\ 0 & 0 & 0 & \left|U_{4}^{test}\right| \end{array}\right] \end{array}$$

where all the off-diagonal elements are zero, $E_{ideal}^{t}\left(i,j\right)=0,i\neq j,\;$indicating no prediction errors. In realistic occasions, all AI models will, no doubt, make errors. Hence, the performance per category is calculated to measure realistic AI models.

RETRACTED

For each class *k* = 1, …, 4, the label of that class is set to *positive*, and the labels of all the rest classes {1, …, *k* − 1, *k* + 1, …, 4} as *negative*. The definitions of true positive (TP), false negative (FN), false positive (FP), and true negative (TN) are illustrated in Figure 8. Three performances metrics (sensitivity, precision, and F1 score) per category are defined:


(33) $$\{\begin{array}{c} Sen\left(k\right)=\frac{TP\left(k\right)}{TP\left(k\right)+FN\left(k\right)}\\ Prc\left(k\right)=\frac{TP\left(k\right)}{TP\left(k\right)+FP\left(k\right)}\\ F1\left(k\right)=\frac{2^{*}Prc\left(z\right)*Sen(z)}{Prc\left(z\right)+Sen(z)} \end{array}\;,k=1,\ldots ,4$$

**Figure 8:** Definition of TP, FN, FP, and TN per category.

The performances of our DFMPNN model are measured over all four categories. The MAF score (symbolized as *F*1_μ_) is harnessed since our dataset is slightly unbalanced. MAF is defined as


(34) $$\begin{array}{l} F1_{\mu }=\frac{2*\mathrm{Pr}c_{\mu }*Sen_{\mu }}{\mathrm{Pr}c_{\mu }+Sen_{\mu }} \end{array}$$

where *Sen*_μ_ and Pr*c*_μ_are defined as.


(35) $$\begin{array}{l} Sen_{\mu }=\frac{\sum_{k=1}^{4}TP\left(k\right)}{\sum_{k=1}^{4}TP\left(k\right)+FN\left(k\right)} \end{array}$$

(36) $$\begin{array}{l} \mathrm{Pr}c_{\mu }=\frac{\sum_{k=1}^{4}TP\left(k\right)}{\sum_{k=1}^{4}TP\left(k\right)+FP\left(k\right)} \end{array}$$

## Experiments, Results, and Discussions

### Parameter Setting

The parameter setting is itemized in Table 6. The STSRs of the four classes are set to 2.27, 2.28, 2.18, and 2.20, respectively. The overall STSR is *m* = 2.23. The width and the height of every image in *F*_*A*_, *F*_*B*_, and *F*_*C*_ are all 1,024. The cropped pixels of all four directions are 200. The final width and the height of the preprocessed image are both 256. The value of DCR is 48. The value of SSR is 97.92%. The number of models in MA is 9. The number of DA is 9. Each DA generates 30 images. The whole augmentation factor is 542. We report our performance on 10 runs over the test set.

**Table 6:** Parameter setting.

**Parameter**	**Value**
$\bar{m}\left(1,2,3,4\right)$	(2.27, 2.28, 2.18, 2.20)
$\bar{m}$	2.23
(*W*_*F*_*A*__, *H*_*F*_*A*__)	(1, 024, 1, 014)
(*W*_*F*_*B*__, *H*_*F*_*B*__)	(1, 024, 1, 014)
(*W*_*F*_*C*__, *H*_*F*_*C*__)	(1, 024, 1, 014)
(*c*_1_, *c*_2_, *c*_3_, *c*_4_)	(200, 200, 200, 200)
(*W*_*F*_*E*__, *H*_*F*_*E*__)	(256, 256)
*v*_*DCR*_	48
*v*_*SSR*_	97.92%
*T*	9
*X*_1_	9
*X*_2_	30
*X*_3_	542
*Q* ^*t*^	10

RETRACTED

### Results of 18-Way DA

Taking Figure 3A as an exemplar raw image *r*(*i*), Figure 9 shows the *X*_1_ different DA results on raw image, i.e., **K**_*x*_[*r*(*i*)], *x* = 1, …, *X*_1_. Due to the page limit, the horizontally mirrored image and its corresponding *X*_1_-way DA results are not shown here.

**Figure 9:** 18-way DA results. **(A)** Image rotation, **(B)** Gaussian noise, **(C)** gamma correction, **(D)** random translation, **(E)** vertical shear, **(F)** salt-and-pepper noise, **(G)** speckle noise, **(H)** horizontal shear, and **(I)** Scaling.

### Confusion Matrix of Our DFMPNN Model

Figure 10 shows the confusion matrix of our DFMPNN model. Five hundred forty-nine are predicted correctly among all the 570 samples of COVID-19, taking the first class as an example. The rest 21 samples, 2, 13, and 6, are wrongly classified as CAP, SPT, and HC, respectively. The measures per category are itemized in Table 7. The sensitivities per class are 96.32, 95.00, 94.92, and 97.21%, respectively. The precisions per class are 94.82, 97.61, 94.75, and 96.42%, respectively. The F1 scores per class are 95.56, 96.29, 94.83, and 96.82%, respectively. Finally, the MAF is 95.88%. Note, in Table 7, the four classes correspond to COVID-19, CAP, SPT, and HC, respectively.

**Figure 10:** Confusion matrix of our DFMPNN model.

**Table 7:** Measures of our DFMPNN model.

**Class**	**Sen**	**Prc**	**F1**
C1	96.32	94.82	95.56
C2	95.00	97.61	96.29
C3	94.92	94.75	94.83
C4	97.21	96.42	96.82
MA			95.88

### Comparison of FMP With Standard Pooling Methods

We now demonstrate the effectiveness of FMP. If we use standard pooling methods with astride of 2, the corresponding networks will shrink faster and have a shallower depth. The three comparison baseline pooling methods are L2-norm pooling (L2P), MP, and AP. The results of 10 runs over the test set are itemized in Table 8.

**Table 8:** Comparison of different pooling methods.

**Model**	**Class**	**Sen**	**Prc**	**F1**	**Model**	**Class**	**Sen**	**Prc**	**F1**
L2P	C1	90.70	91.50	91.10	MP	C1	91.58	92.23	91.90
	C2	90.18	89.38	89.78		C2	91.25	92.57	91.91
	C3	93.22	94.18	93.70		C3	93.56	91.85	92.70
	C4	92.95	92.05	92.50		C4	95.08	94.93	95.00
	MA			91.80		MA			92.92
AP	C1	90.53	93.14	91.81	FMP (Ours)	C1	96.32	94.82	95.56
	C2	93.39	93.06	93.23		C2	95.00	97.61	96.29
	C3	92.54	91.76	92.15		C3	94.92	94.75	94.83
	C4	93.61	92.25	92.92		C4	97.21	96.42	96.82
	MA			92.53		MA			95.88

The bar plot is shown in Figure 11, where *k*−*S, k*−*P, k*−*F, and k* ∈ {1, 2, 3, *and* 4} stand for the sensitivity, precision, and F1 score for category *k*. The rightmost bar “MAF” stands for the micro-averaged F1 score. In terms of MAF, our DFMPNN model based on FMP attains the best results of 95.88%. The second best is MP, with an MAF of 92.92%. The AP ranks the third best with an MAF of 92.53%. The worst is L2P, with an MAF of 91.80%.

RETRACTED

**Figure 11:** A 3D bar plot of SPNN vs. other pooling methods.

The reason why our FMP attains the best results are two points: (i) The FMP makes the reduction of FM slower, so it can create a deeper network. (ii) The MA helps recreate the performance of our DFMPNN network. In the future, we shall try two FMP extension models (27, 28) to test whether we can further the performances.

### Comparison to State-of-the-Art Models

We compared our proposed DFMPNN method with 10 state-of-the-art methods: WEBBO (8), 3SBBO (9), DeCovNet (10), FSVC (11), GN-COD (12), GLCMSVM (13), 5L-DCNN (14), CSSN (15), FCONet (16), COVNet (17). All the comparison was carried on over the same test set of 10 runs. The comparison results are itemized in Table 9.

**Table 9:** Comparison with state-of-the-art models.

**Model**	**Class**	**Sen**	**Prc**	**F1**	**Model**	**Class**	**Sen**	**Prc**	**F1**
WEBBO (8)	C1	76.49	76.22	76.36	3SBBO (9)	C1	82.63	83.96	83.29
	C2	72.50	71.60	72.05		C2	80.89	76.26	78.51
	C3	74.07	72.59	73.32		C3	84.58	85.15	84.86
	C4	71.31	73.85	72.56		C4	81.15	84.04	82.57
	MA			73.56		MA			82.32
DeCovNet (10)	C1	91.05	90.58	90.81	FSVC (11)	C1	91.40	90.14	90.77
	C2	93.75	90.99	92.35		C2	87.32	86.55	86.93
	C3	90.51	86.97	88.70		C3	91.19	91.03	91.11
	C4	88.69	95.58	92.01		C4	90.16	92.28	91.21
	MA			90.94		MA			90.04
GN-COD (12)	C1	83.68	83.10	83.39	GLCMSVM (13)	C1	68.07	68.55	68.31
	C2	85.36	83.86	84.60		C2	72.14	71.25	71.69
	C3	88.31	90.29	89.29		C3	71.02	70.9	70.96
	C4	85.08	85.22	85.15		C4	83.44	83.99	83.72
	MA			85.62		MA			73.82
5L-DCNN (14)	C1	93.16	91.39	92.27	CSSN (15)	C1	94.04	92.25	93.14
	C2	93.21	91.10	92.14		C2	93.75	95.11	94.42
	C3	91.53	91.53	91.53		C3	91.36	93.58	92.45
	C4	86.56	90.10	88.29		C4	94.43	92.75	93.58
	MA			91.03		MA			93.39
FCONet (16)	C1	92.28	95.64	93.93	COVNet (17)	C1	89.82	86.63	88.20
	C2	96.79	94.43	95.59		C2	89.82	92.63	91.21
	C3	94.75	95.88	95.31		C3	93.73	90.66	92.17
	C4	94.92	92.94	93.92		C4	87.38	90.96	89.13
	MA			94.68		MA			90.17
DFMPNN (Ours)	C1	96.32	94.82	95.56					
	C2	95.00	97.61	96.29					
	C3	94.92	94.75	94.83					
	C4	97.21	96.42	96.82					
	MA			95.88					

Figure 12 compares the proposed DFMPNN model with 10 state-of-the-art models. All the models are ranked by the MAF performance (last column in Figure 12) in a descending direction. We can observe from Figure 12 that the proposed DFMPNN achieves the highest MAF value among all algorithms.

RETRACTED

**Figure 12:** A 3D bar plot of algorithm comparison.

## Conclusion

We not only propose a DFMPNN model but also integrate three improvements: (i) The FMP replaces traditional MP and AP. (ii) Multiple-way DA is utilized. (iii) DFMPNN is proven to yield better results than 10 state-of-the-art models.

The shortcomings of this model are four points. First, some advanced AI modules are not integrated, which may help improve the performance. Second, more advanced pooling techniques could be tested. Third, the dataset is relatively small. Fourth, we do not have an environment to clinically validate our model.

To solve those weak points, we shall try to integrate more advanced DL modules, such as graph networks, attention mechanisms, etc. Meanwhile, some advanced pooling techniques will be tested, such as stochastic pooling, rank-based pooling, etc. Furthermore, we shall try to combine several COVID-19 datasets from different resources so as to make our model tested on more datasets. Finally, we shall try to distribute our software to hospital staff, and let them test the proposed model.

## Data Availability Statement

The dataset is available upon reasonable request to corresponding authors. Requests to access these datasets should be directed to Yu-Dong Zhang, yudongzhang@ieee.org.

## Author Contributions

S-HW: conceptualization, software, formal analysis, methodology, writing, review, editing, visualization, and funding acquisition. SS: methodology, writing—original draft, project administration, and resources. DA: writing—original draft, writing, review, editing. S-XC: data curation, writing—original draft, writing, review, editing, project administration, and supervision. Y-DZ: conceptualization, methodology, resources, writing—original draft, writing, review, and editing, visualization, project administration, supervision, and funding acquisition. All authors contributed to the article and approved the submitted version.

## Conflict of Interest

The authors declare that the research was conducted in the absence of any commercial or financial relationships that could be construed as a potential conflict of interest.

## Publisher's Note

All claims expressed in this article are solely those of the authors and do not necessarily represent those of their affiliated organizations, or those of the publisher, the editors and the reviewers. Any product that may be evaluated in this article, or claim that may be made by its manufacturer, is not guaranteed or endorsed by the publisher.
